The article "Credit Risk Evaluation of Asset Securitization of PPP Project of Sports Public Service Venues Based on Random Forest Algorithm" was published in 2022. Journal: Comput Intell Neurosci.

# Credit Risk Evaluation of Asset Securitization of PPP Project of Sports Public Service Venues Based on Random Forest Algorithm

**DOI:** 10.1155/2022/5177015

**Published:** 2022-08-08

**Authors:** Yanshou Wang

**Affiliations:** ^1^School of Economics and Management, Shanghai University of Sport, Shanghai, China; ^2^Sports Economics Management Research Center, Shanghai University of Engineering Science, Shanghai, China

## Abstract

Due to the characteristics of sports public service venues, there are still some financing difficulties under the PPP (public-private partnership) operation mode. Although asset securitization can solve its corresponding problems and enhance the standardization of PPP projects, its many participants, complex transaction structure, and other influencing factors still have a great impact on the financing effect. Therefore, this paper integrates the random forest algorithm into the asset securitization credit risk evaluation system of PPP project of sports public service venues, and screens the audition indicators of credit risk evaluation through the constructed model. The experimental results show that optimizing the parameter setting of random forest model can effectively reduce the misjudgment rate of default samples, while maintaining the stability of other performance indicators. Even if other misjudgment rates will increase to a certain extent, it is within a reasonable range, which improves the overall performance of the model. The ROC curve shows that the risk credit indicators selected by the model have strong evaluation performance and effectiveness and can provide some reference information for the credit risk prevention of asset securitization of PPP project of sports public service venues.

## 1. Introduction

The improvement of national fitness awareness is one of the important driving forces for the development of sports industry. More different types of sports have gradually entered public life. People's demand for sports venues has also changed from simplification to diversification and specialization. The construction of sports public service venues has entered a stage of rapid development [1]. For any country or city, hosting large-scale sports events, especially international sports events, can promote economic development, promote the adjustment of economic structure and the solution of social employment and other problems, and improve the popularity of countries and cities. Similarly, countries and cities that can host large-scale sports events also show certain advantages in terms of infrastructure, environmental conditions, comprehensive strength, and event experience [2]. However, with the development of sports events, the infrastructure and stadiums established in the past cannot meet the needs of more and more professional sports events. The stadiums and gymnasiums operated by the government after the game cannot produce good social benefits and even become idle buildings because of the single function, low actual utilization rate and the operation mode do not meet the market demand. This situation undoubtedly increases the financial burden of the local government and fails to achieve the purpose of making full use of social resources [3]. Therefore, combined with past cases and experience, the construction and management of sports public service venues has produced a form of cooperation between the government and social capital, namely PPP mode. With the participation of the government, it actively absorbs social capital, separates the ownership and management right of sports public service venues, and produces various types of cooperation modes [4]. Therefore, the research in this paper study PPP project, it as a new financing mode of sports public service venues, PPP mode has obvious effect in reducing the financial pressure of the government in the early stage of development and promoted the development process of public utilities. On the other hand, during the development of PPP projects, problems such as difficult financing and difficult withdrawal of social capital have gradually emerged. These problems existing in the PPP project of sports public service venues can be solved to a great extent by means of asset securitization, which is also the new direction and new road of its development.

The article "Credit Risk Evaluation of Asset Securitization of PPP Project of Sports Public Service Venues Based on Random Forest Algorithm" was published in 2022. Journal: Comput Intell Neurosci.

Basic assets are an important foundation and guarantee for the realization of asset securitization of PPP projects. Asset securitization can improve the standardization of PPP projects and reduce the difficulty of financing [5]. However, the PPP project of sports public service venues itself has a long life cycle, many participants, and complex transaction relations. Therefore, there are many risk factors that will affect the asset securitization of the project [6]. The credit of assets is the foundation for PPP projects to realize asset securitization and promote project development. Based on the random forest algorithm, this paper constructs the credit risk evaluation model and the corresponding credit risk evaluation index system of asset securitization of PPP project of sports public service venues, verifies the evaluation model through empirical analysis, and analyzes the results.

## 2. Research Status of Asset Securitization of PPP Projects at Home and Abroad

PPP mode was initially emerging abroad. Many scholars have studied the risk and possibility of projects operated through this mode. Some scholars have analyzed the risk-taking mechanism of PPP model from the perspective of macrosystem, microsystem, and private sector, and pointed out that there are differences in risk types of different PPP projects [7]. As for the necessary conditions for asset securitization to achieve the purpose of financing, some scholars believe that this method can reduce the financing cost of sponsors and stimulate the enthusiasm of investors and the degree of market participation [8]. Some scholars also pointed out that asset securitization is the process of transforming fixed assets into securities, and the process of transforming illiquid assets into valuable investment, which can promote market liquidity. Similarly, it has a certain demand for the market environment [9]. Therefore, for the asset securitization of PPP projects, some scholars pointed out that asset securitization is an important means to improve the liquidity and profitability of PPP projects [10]. Other scholars have concluded through corresponding research that PPP projects can effectively reduce financing costs through asset securitization, and its financing effect will be affected by environmental factors such as government and public support [11].

The article "Credit Risk Evaluation of Asset Securitization of PPP Project of Sports Public Service Venues Based on Random Forest Algorithm" was published in 2022. Journal: Comput Intell Neurosci.

Relatively speaking, the development of domestic PPP mode started late and there are relatively few examples that can be studied. The research in many aspects, such as project feasibility, impact and prevention of risk factors, is still in the exploratory stage [12]. Some scholars concluded through analysis that the risks of PPP project itself, the risks of all participants and the risk of benefit distribution need to be analyzed and prevented. At the same time, the project contract risks, especially the terms of franchise rights, need to be paid attention to [13]. Some scholars studied the credit enhancement system of asset securitization and pointed out that the effect of the current credit enhancement system in reducing credit risk is not ideal, and the system needs further improvement [14]. Other scholars put forward suggestions beneficial to the progress of asset securitization of domestic PPP projects based on the WBS financing model experience of Britain and the United States [15]. According to the domestic urban construction process, some scholars believe that the development of asset securitization of PPP project meets the needs of urban construction and development. It can meet the needs of a large number of infrastructure and public construction, relieve the pressure of government funds, reduce project financing risks, and broaden financing channels [16].

## 3. Construction of Credit Risk Assessment Model for Asset Securitization of PPP Project of Sports Public Service Venues Based on Random Forest Algorithm

### 3.1. Feasibility of Asset Securitization of PPP Project of Sports Public Service Venues

Firstly, the realization of asset securitization of PPP project of sports public service venues needs the support of relevant policies. In the released policy document, it is pointed out that while reducing the high debt ratio of state-owned enterprises, it is necessary to provide good policies and create a good institutional environment, encourage the absorption and supplement of social capital according to law, broaden the channels of equity financing, inject new capital vitality into the stock assets of state-owned enterprises, maximize the benefits of existing resources, and provide a strong driving force for the virtuous circle development of sports industry [17]. By virtue of the communication and cooperation mechanism, diversified investment and financing subjects can increase communication channels and obtain more relevant information, reduce the operation risk of sports public service venues, improve their operation efficiency, and promote the process of asset securitization of the project [18].

The article "Credit Risk Evaluation of Asset Securitization of PPP Project of Sports Public Service Venues Based on Random Forest Algorithm" was published in 2022. Journal: Comput Intell Neurosci.

Secondly, social capital provides the original capital for the asset securitization transformation of PPP projects of sports public service venues. Social capital includes idle funds owned by residents and large-scale savings funds, and their huge investment benefits have not been brought into full play [19]. Sports public service venues need capital accumulation, and the existence of social capital provides them with the possibility and conditions to complete capital accumulation [20].

Finally, the asset securitization transformation of PPP project of sports public service venues meets the market demand. Project asset securitization effectively reduces the dependence of stadiums and gymnasiums on government and state-owned funds. At the same time, sports public service stadiums and gymnasiums have good reputation and are guaranteed by future income and government tax, which increases their securitization credit and reduces investment risk [21]. The process of project asset securitization is also the embodiment of realizing the economic and social benefits of venues, which can play its potential functional value [22].

As shown in Figure 1, it is the asset securitization process and corresponding subjects of PPP project of sports public service venues.

### 3.2. Audition and Data Processing of Credit Risk Assessment Index System for Asset Securitization of PPP Project

Compared with the general project asset securitization, the PPP project asset securitization of sports public service venues has a long cycle, complex links, and diversified participants. A credit crisis in any link will damage the securitization quality of the whole project. Therefore, the credit risk of project asset securitization is the most concerned link of investment participants. The audition of the evaluation index system is carried out according to the characteristics of sports public service venues, the credit indicators of Galway at home and abroad, and the index system sorted out in relevant literature research. Its credit risk mainly comes from the credit risk of each participant in the process of securitization, government credit risk, basic asset credit risk of PPP project of sports public service venues, and transaction structure credit risk, which is used as the criterion level to build an audition index set [23].

The article "Credit Risk Evaluation of Asset Securitization of PPP Project of Sports Public Service Venues Based on Random Forest Algorithm" was published in 2022. Journal: Comput Intell Neurosci.

In order to ensure the standardization and unity of a large amount of relevant index data, data preprocessing measures need to be taken to prepare for the screening of indicators in random forest model. The data standardization processing is shown in equations (1)–(3).

Standardized equation of positive credit evaluation index:

(1) $$\begin{array}{c} y_{mn}=\frac{x_{mn}-\min_{1\leq m\leq q}x_{mn}}{{\text{max}}_{1\leq m\leq q}x_{mn}-\min_{1\leq m\leq q}x_{mn}}. \end{array}$$

Standardized equation of negative credit evaluation index:

(2) $$\begin{array}{c} y_{mn}=\frac{\min_{1\leq m\leq q}x_{mn}-x_{mn}}{\max_{1\leq m\leq q}x_{mn}-\min_{1\leq m\leq q}x_{mn}}. \end{array}$$

Standardized equation of interval credit evaluation index:

(3) $$\begin{array}{c} y_{mn}=\left\{\begin{array}{cc} 1-\;\frac{a_{1}-x_{mn}}{\max\left(a_{1}-\min\left(x_{mn}\right),\max_{1\leq m\leq q}\left(x_{mn}\right)-a_{2}\right)}, & x_{mn}<a_{1},\\ 1-\frac{x_{mn}-a_{2}}{\max\left(a_{1}-\min\left(x_{mn}\right),\max_{1\leq m\leq q}\left(x_{mn}\right)-a_{2}\right)}, & x_{mn}>a_{2},\\ 1, & a_{1}\leq x_{mn}\leq a_{2}. \end{array}\right) \end{array}$$

### 3.3. Principle of Credit Risk Assessment System for Asset Securitization of PPP Project Based on Stochastic Forest Algorithm

The unit classifier of random forest algorithm is cart classification tree and contains multiple classification trees. Each classification tree corresponds to a training subset formed by independent sampling and maintains the same index selection probability, which is repeated constantly [24]. The results of these classification trees are different and independent of each other, and then the final classification results are selected by simple voting on the results of the classification tree [25]. As shown in Figure 2, the establishment flowchart of index system based on random forest algorithm is shown.

The article "Credit Risk Evaluation of Asset Securitization of PPP Project of Sports Public Service Venues Based on Random Forest Algorithm" was published in 2022. Journal: Comput Intell Neurosci.

The cart classification tree in the random forest model is like a tree, which contains three nodes: root, middle, and leaf. The root node is the place where all sample data are input. The input samples have the same number of index attributes, and these index attributes form a candidate index set to be divided. After traversing each index attribute, there is and only one selection opportunity. In the middle part of the node, the optimal classification index and corresponding value selected in the sample are divided according to the Gini coefficient principle, and the cycle operation is carried out until all the samples contained in the leaf node belong to the same class. At this time, the candidate index set is empty, and if it is satisfied at the same time, the segmentation stops. Let *T* represent the node before segmentation, *t*_1_, *t*_2_ is the node after segmentation, the classification type represents *Y*, the number of sample types contained in *T* is *j*, and the probability of a category in the node after segmentation is represented by *P*(*Y*_*n*_ *|* *t*_*m*_). When the split point is selected as a specific value in the index, the Gini index of the split node *t*_*m*_ is calculated as shown in the following:

(4) $$\begin{array}{c} \text{Gini}\left(t_{m}\right)=1-\sum_{n=1}^{2}{\left[P\left(Y_{n}\;|\;t_{m}\right)\right]}^{2}. \end{array}$$

The above indicates that when the segmentation node contains only the same type of samples, the Gini index reaches the minimum value. When the segmentation node contains different types of samples with the same proportion, the Gini index reaches the maximum.

The Gini impure of any index attribute divided by the node can be calculated by

(5) $$\begin{array}{c} \text{Gini}\left(T\right)=\sum_{m=1}^{2}\frac{i_{m}}{i}\text{Gini}\left(t_{m}\right), \end{array}$$

where the number of split nodes is *m*, the number of samples in the split node is *i*_*m*_, and *i* represents the total number of samples in the node.

The independent sampling of cart classification tree is a random sampling operation with return, so the probability of each sampling is equal to each sample, all 1/*i*, and the *i* probability of not being selected in the second sampling is shown in the following:

(6) $$\begin{array}{c} P={\left(1-\frac{1}{i}\right)}^{i}. \end{array}$$

If the number of original samples in the above equation is sufficient, the probability value will gradually converge. The convergence value is 1/*e*, that is, only nearly 63.2% of the samples in the sample set may exist in the training subset, and the nonexistent part belongs to “out-of-bag data,” that is, OOB.

The article "Credit Risk Evaluation of Asset Securitization of PPP Project of Sports Public Service Venues Based on Random Forest Algorithm" was published in 2022. Journal: Comput Intell Neurosci.

After the construction of random forest model is completed, its prediction estimation is completed through OOB, and its accuracy estimation is shown in the following:

(7) $$\begin{array}{c} Q_{m}\left(x,y\right)=\frac{\sum_{m=1}^{k}I\left(h_{m}\left(x\right)=y,\left(x,y\right)\in O_{m}\left(x\right)\right)}{\sum_{m=1}^{k}I\left(h_{m}\left(x\right),\left(x,y\right)\in O_{m}\left(x\right)\right)}. \end{array}$$

The denominator in the above equation is the total number of samples that have not been drawn, and the numerator is the number of correctly classified samples that have not been drawn.

The prediction result of each classification tree represents a type vote, and the category with the highest number of votes is the prediction classification label. For example, (8) represents the calculation of prediction result:

(8) $$\begin{array}{c} Y_{f}=\text{arg}\underset{y}{\max}\sum_{k=1}^{n\text{tree}}\delta \left(h\left(x,\theta_{k}\right)=y\right), \end{array}$$

where *n*tree represents the number of decision trees and *δ*(•) represents the indicative function.

The generalization error obtained from the OOB input model can effectively measure the classification performance of the model. The interval function and the mathematical expression of generalization error are shown in the following:

(9) $$\begin{array}{c} mg\left(x,y\right)=ave_{k}\delta \left(h_{k}\left(x\right)=y\right)-\underset{n\neq y}{{\text{max ave}}_{k}\delta \left(h_{k}\left(x\right)=n\right)}, \end{array}$$

(10) $$\begin{array}{c} Pe^{*}=P_{x,y}\left(mg\left(x,y\right)<0\right). \end{array}$$

In the equation, the average value of the sample correctly predicted with label *y* is expressed as ave_*k*_*δ*(*h*_*k*_(*x*)=*y*), and the maximum average value of the sample not predicted with label *y* is expressed as maxave_*k*_*δ*(*h*_*k*_(*x*)=*n*)_*n*≠*y*_; *Pe*^*∗*^ is the generalization error.

In the form of interval function, its edge function can be defined as shown in the following:

(11) $$\begin{array}{c} mr\left(x,y\right)=P\left(h_{m}\left(x\right)=y\right)-\underset{n\neq y}{\max}\left\{P\left(h_{m}\left(x\right)=n\right)\right\}. \end{array}$$

In the equation, the probability represented by *P*(*h*_*m*_(*x*)=*y*) is the probability of correct judgment, and max_*n*≠*y*_{*P*(*h*_*m*_(*x*)=*n*) is the maximum probability of incorrect judgment.

As shown in Figure 3, the confusion matrix of the evaluation index of random forest algorithm is divided into two categories: nondefault samples, i.e., 0. Otherwise, it is default samples, i.e., 1. The number of correctly predicted nondefault samples is expressed as TP. The number of default samples correctly predicted is expressed as TN. The number of prediction result errors in the nondefault sample is FN. The number of prediction errors in the default sample is FP.

The article "Credit Risk Evaluation of Asset Securitization of PPP Project of Sports Public Service Venues Based on Random Forest Algorithm" was published in 2022. Journal: Comput Intell Neurosci.

The sensitivity of random forest model is calculated according to

(12) $$\begin{array}{c} \text{TPR}=\frac{\text{TP}}{\left(\text{TP}+\text{FN}\right)}\text{.} \end{array}$$

The specificity calculation equation is shown in the equation:

(13) $$\begin{array}{c} \text{TNR}=\frac{\text{TN}}{\left(\text{TN}+\text{FP}\right)}. \end{array}$$

The accuracy is calculated by:

(14) $$\begin{array}{c} \text{precision}=\frac{\text{TP}}{\left(\text{TP}+\text{FP}\right)}. \end{array}$$

The accuracy calculation is shown in the following:

(15) $$\begin{array}{c} \text{ACC}=\frac{\left(\text{TP}+\text{TN}\right)}{\left(\text{TP}+\text{FN}+\text{TN}+\text{FP}\right)}. \end{array}$$

The error rate calculation equation is:

(16) $$\begin{array}{c} E=1-\text{ACC}. \end{array}$$

By introducing the influence of random noise into the random forest model, the importance level of credit evaluation indicators can be determined by the change of prediction accuracy. The calculation equation is shown in the following:

(17) $$\begin{array}{c} {\text{DIFF}}_{m}=\frac{\text{ACC}-\sum_{k=1}^{n\text{tree}}{\text{ACC}}_{km}}{n\text{tree}}. \end{array}$$

where ACC_*km*_ represents the OOB estimation accuracy of *k* classification tree after all out-of-bag sample values of index attribute *m* in random order.

The weight value of credit risk evaluation index is calculated according to

(18) $$\begin{array}{c} w_{m}=\frac{{\text{DIFF}}_{m}}{\sum_{m=1}^{M}{\text{DIFF}}_{m}}. \end{array}$$

The weight value is expressed as *w*_*m*_ and the number of credit risk assessment indicators of asset securitization is expressed as *M*.

On this basis, the index importance level and its relationship of random forest algorithm are reflected by

(19) $$\begin{array}{c} E{\left(C\right)}_{m}=\sum_{n=1}^{M}\left[\left(y_{\left(mn\right)}-y_{\left(mn-1\right)}\right)w_{n}\right], \end{array}$$

where *E*(*C*)_*m*_ represents the credit evaluation score, *y*_(*mn*)_ is the standard value of the *n* credit evaluation index of *m*, and *w*_*n*_ is the weight value. The credit rating range (as shown in (1) and (20)) needs to be converted to the credit rating range of [1, 20]:

(20) $$\begin{array}{c} Z_{m}=\frac{E_{m}-\text{min}\left(E_{m}\right)}{\max\left(E_{m}\right)-\text{min}\left(E_{m}\right)}\times 100. \end{array}$$

## 4. Empirical Analysis on Credit Risk Assessment of Asset Securitization of PPP Project of Sports Public Service Venues Based on Random Forest Algorithm

The contract term of a large-scale sports public service venue PPP project is 25 years. According to the relevant contracts, the project company is responsible for the construction of sports public service venues, has the right to operate sports public service venues, and is responsible for their operation, daily maintenance, venue transformation, and renewal. During the contract period, the venue shall provide the government with event services that meet the event standards, and the project company shall ensure the integrity and good operation of the stadium. According to the characteristics of the project, the audition indicators of asset securitization credit risk of the project were shown in Table 1.

The article "Credit Risk Evaluation of Asset Securitization of PPP Project of Sports Public Service Venues Based on Random Forest Algorithm" was published in 2022. Journal: Comput Intell Neurosci.

After data preprocessing and standardization, 70% of the credit evaluation samples are randomly selected as the training set and the rest are the test set. Random forest algorithm will produce different results due to the difference of many parameter settings. In order to reduce the subjectivity of parameter settings, it will be analyzed through two aspects: model selection characteristics and decision tree. As shown in Figure 4, the relationship between the number of different decision trees and OOB error when the range of feature numbers is determined. It can be concluded that the model OOB error does not change monotonically with the increase of the number of selected features, but shows a fluctuating state. Similarly, the OOB error does not decrease with the increase of the number of decision trees. Relatively speaking, when the number of selection features is four and the number of decision trees is 100, the OOB error appears local minimum.

In this case, let the maximum feature number be four, and analyze the OOB error of the number of decision trees from 80 to 120. As shown in Figure 5, when the number of decision trees is 105, the OOB error value reaches the minimum.

As shown in Figure 6, it is a scatter diagram between the mtry parameter of the model and the OOB misjudgment rate of the model. The larger the mtry parameter, the greater the OOB misjudgment rate. When it reaches 38, the misjudgment rate tends to converge and fluctuates in a small range. Therefore, the optimal value of the parameter mtry is 1.

In order to confirm the rationality of parameter setting and model optimization, the judgment results of the model with default parameters and optimized parameters are compared, and the results are shown in Figure 7. The comparison results show that under the default parameters, the misjudgment rate of default samples is higher, and the misjudgment rate can be effectively reduced by optimizing the parameter settings. While other evaluation indicators remain in a high state after optimization, and the increase of some indicators is also within a reasonable range, so the optimization of model parameters is reasonable.

The article "Credit Risk Evaluation of Asset Securitization of PPP Project of Sports Public Service Venues Based on Random Forest Algorithm" was published in 2022. Journal: Comput Intell Neurosci.

Further verify the effectiveness of the risk assessment module analysis results, and randomly select samples different from the original sample set for judgment, as shown in Figure 8. The data showed that the model evaluation index results obtained after the optimization of the randomly selected sample set are high, and the misjudgment rate remains low, which meets the requirements of index screening.

Keep one of the repeated indicators in the audition indicators, and then randomly select three different sample sets for the same parameter setting optimization to screen the remaining credit risk evaluation indicators. The indicators that appear repeatedly in the model results are selected as the final credit risk evaluation indicators.  Figure 9 shows the final credit risk evaluation indicators and their importance distribution. The results show that the effectiveness of the measures of bankruptcy isolation in the process of asset securitization of the PPP project of sports public service venues is weak.

As shown in Figure 10, the ROC curve of the random forest model in this paper can reflect the effectiveness of the model. There is a large area below the curve in the figure, which means that the credit risk index system in this paper has strong evaluation performance and high effectiveness for the credit risk of asset securitization of PPP project of sports public service venues.

## 5. Conclusion

In the previous years, sports public service venues were mainly funded and operated and managed by the government. However, because the management mode could not keep up with the market demand, the single venue function could not meet the diversified needs of the public and many venues could not operate normally, while increasing the financial burden. PPP mode could use social funds to alleviate the pressure of government funds, improve the operation and management ability of venues, and follow the development of market demand. However, this model was still in its infancy, the system standardization was relatively low, and there were still many problems. Asset securitization can improve the standardization of PPP projects, reduce financing costs, and provide more guarantee for the development of sports public service venues. This paper introduces the stochastic forest model into the credit risk system of asset securitization of PPP project, and constructs the corresponding evaluation index. The experimental results show that the credit risk evaluation model based on random forest algorithm can maintain high model performance indicators, reduce the misjudgment rate of default samples, and improve the overall performance of the model. The credit risk indicators selected by the model have strong evaluation performance and high effectiveness for the credit risk of asset securitization of PPP project of sports public service venues. The random forest model constructed in this paper still has shortcomings and its performance in the extended data set needs to be verified. At the same time, the process of asset securitization of PPP project of sports public service venues involves many links. The influencing factors studied in this paper are limited and need to be further expanded.

The article "Credit Risk Evaluation of Asset Securitization of PPP Project of Sports Public Service Venues Based on Random Forest Algorithm" was published in 2022. Journal: Comput Intell Neurosci.

## Figures and Tables

**Figure 1:** Asset securitization process and corresponding subjects of PPP project of sports public service venues.

**Figure 2:** Flowchart of establishing index system based on random forest algorithm.

**Figure 3:** Confusion matrix of evaluation index of random forest algorithm.

**Figure 4:** The relationship between the number of different decision trees and OOB error when the range of characteristic numbers is determined.

**Figure 5:** When the maximum feature number is determined, the number of different decision trees and OOB error.

**Figure 6:** Scatter plot between model mtry parameters and model OOB misjudgment rate.

**Figure 7:** Comparison of model judgment results of default parameters and optimized parameters.

**Figure 8:** Another randomly selected different sample judgment results.

**Figure 9:** Final credit risk evaluation index and its importance distribution.

**Figure 10:** ROC curve of random forest model.

**Table 1:** Audition indicators of credit risk of project asset securitization.

First level criterion layer	Secondary criterion layer	Index layer
Credit risk of each participant	Credit risk of original equity holders/asset service institutions	X1 asset structure X2 liability structure X3 solvency X4 profitability X5 cash flow X6 main business X7 growth capability X8 operating capacity X9 conflict of contract documents X10 service quality X11 changes in market demand X12 operation change risk
	Credit risk of plan manager	X13 risk coverage X14 capital leverage ratio X15 liquidity coverage X16 net stable capital ratio
	Credit risk of difference payment commitment	X17 financial data X18 cash flow
	Credit rating risk	X19 credit rating risk X20 rating agency

Credit risk of project underlying assets	Quality risk of underlying assets	Construction of x21 ppp project X22 profit model X23 construction quality X24 project approval delay X25 financing risk
	Cash flow forecast risk of underlying assets	X26 historical government payment X27 cash flow forecast X28 cash flow coverage X29 cash flow forecast deviation risk X30 credit enhancement method X31 legal ownership risk of underlying assets

Transaction structure credit risk	—	X32 real sale risk of underlying assets
		X33 spv bankruptcy risk
		X34 risk of fund mixing and misappropriation

Government credit risk	—	X35 government performance risk X36 government deferred payment risk X37 government prepayment risk X38 government decision risk X39 perfection of relevant laws X40 perfection of supervision system

The article "Credit Risk Evaluation of Asset Securitization of PPP Project of Sports Public Service Venues Based on Random Forest Algorithm" was published in 2022. Journal: Comput Intell Neurosci.

## Data Availability

All data used to support the findings of this study are included within this article.
